The article "Efficacy and Safety of Rituximab in the Treatment of Idiopathic Membranous Nephropathy: A Meta-Analysis" was retracted in 2023. Reasons: signs of a paper mill; suspected computer-generated content; unreliable results or conclusions; concerns about the data.

# Efficacy and Safety of Rituximab in the Treatment of Idiopathic Membranous Nephropathy: A Meta-Analysis

**DOI:** 10.1155/2022/5393797

**Published:** 2022-10-12

**Authors:** Huijuan Lu, Jun Shen, Jieqiong Sun, Jia Sun

**Affiliations:** Department of Nephrology, First People's Hospital of Linping District, No. 369, Yingbin Road, Linping District, Hangzhou, Zhejiang 311199, China

## Abstract

**Background:**

Primary membranous nephropathy (MN), sometimes referred to as idiopathic membranous nephropathy (IMN), is a kind of MN whose pathogenesis is yet unclear. According to research reports, the incidence of IMN is about 9.8–26.8%, and it is on the rise.

**Methods:**

The computer retrieves eight databases to obtain controlled trials at home and abroad on the rituximab (RTX) actions in IMN management. After a rigorous literature quality evaluation, software called RevMan 5.3 was used for data analysis.

**Results:**

This meta-analysis finally contained 8 papers. They were all regarded as controlled trials. Six studies reported serum creatinine (standardized mean difference [SMD]: −6.87; 95% CI: −14.09, 0.35; *P* = 0.062), ALB (SMD: 1.91; 95% CI: −0.31, 4.14; *P* = 0.092), and adverse reactions (OR: 0.56; 95% CI: 0.36, 0.90; *P* < 0.01), all of which were significantly higher in the test group than in the control group (OR: 1.37; 95% CI: 1.07, 1.76; *P* < 0.01)

**Conclusion:**

The overall effective rate, serum creatinine, adverse effects, and ALB of this trial indicate that RTX may be beneficial for individuals with IMN, but further high-quality research is required to confirm these findings.

## 1. Introduction

Primary membranous nephropathy (MN), commonly known as idiopathic membranous nephropathy (IMN), is a type of MN whose pathogenesis is yet unclear. MN is a non-inflammatory mediated autoimmune disease, which is characterized by the deposition of immune complexes formed by autoantibodies in the glomerular basement membrane, causing thickening and stiffness of the glomerular basement membrane, and also leading to renal disease in adults, which is one of the main causes of the syndrome [14]. Epidemiological surveys in recent years have found that the incidence of MN in China has increased from 9.8 to 26.8%, and it has become one of the important causes affecting the health of Chinese residents [15–17]. The bulbar foundation membrane thickens diffusely, which is one of its characteristics. Individuals with clinical signs of nephrotic syndrome (large proteinuria, hypoproteinemia, edema, and hyperlipidemia) accounts for 80% of cases. Investigations [1] have shown that the incidence of IMN is increasing at a rate of 13% year by year, which may be related to factors such as increasing environmental pollution and increased prevalence of metabolic diseases. There are several IMN prognosis. Around 1/3 of sufferers in the clinic can have spontaneous remission, and 40% of the patients continue to progress and worsen and eventually develop into chronic renal failure. Age, gender, baseline glomerular filtration rate decline, urinary small molecular protein components, such as *β*2 microglobulin and anti-phospholipase A2 receptor (PLA2R) level after treatment may be correlated with prognosis.

MN is divided into secondary membranous nephropathy (SMN) and IMN according to the etiology. About 20% of patients with MN have systemic causes, such as autoimmune diseases, infections and tumors, or are exposed to certain factors, such as drugs and poisons which are called as SMN. 80% of patients with MN are limited to kidney involvement, which is called IMN due to the unclear etiology. In recent years, it has been found that the PLA2R and type 1 thrombospondin 7A domain (thrombospondin type 1 domain-containing 7A, THSD7A) is one of the target antigens of autoantibodies and the main cause of IMN. About 70% of IMN patients have positive serum anti-PLA2R antibodies, while about 20% of negative patients are THSD7A-positive [18–23].

At the moment, kidney biopsy pathology is the mainstay of the IMN diagnosis. For the confirmed patients, the disease must first be evaluated to determine the risk of disease progression. Generally, non-specific supportive treatment is required first, and specific immunotherapy can be started for those with medium and high risk. For IMN patients who need to receive immunosuppressive therapy, there are many types of immunosuppressive agents available, including glucocorticoids, alkylating agents, and calcineurin inhibitors [2].

Although IMN is considered a “benign disease,” the renal function of patients is often stable for a long time, and about one-third of patients with MN can experience spontaneous remission of the disease after the discovery of MN, but there are still 30–40% of IMN patients, especially those with persistent massive proteinuria or decreased renal function, tend to be prone to gradual progression to end-stage renal disease over 5–15 years [3–5]. Although the KDIGO guidelines have recommended the treatment of IMN, the treatment of IMN is still controversial [6]. At present, IMN is considered to be an autoimmune disease, and studies have found that the activation of immune pathways in the glomerulus can lead to renal damage and renal function progression [7], so immunosuppressive therapy may be a reasonable choice. But due to immune, the significant side effects of inhibitor use and the phenomenon of spontaneous remission in IMN patients are particularly important to select appropriate treatment targets. In recent years, with the rapid development of precision medicine, the use of existing clinical data and appropriate model construction methods to construct accurate prognosis prediction models will help to screen suitable treatment targets. Previous studies have found that massive proteinuria, renal impairment, gender, blood pressure, and age are closely related to the renal prognosis of IMN patients, and some studies have suggested that the serum anti-PLA2R antibody concentration is also one of the important indicators to predict the prognosis of IMN patients [8–13].

Rituximab (RTX), a chimeric monoclonal antibody made by genetic engineering of human and murine cells, hits the CD20 antigen on the membrane of B lymphocytes and prevents their proliferation and development. It prevents the proliferation and development of B cells by concentrating on the CD20 antigen on the membrane of B lymphocytes. In clinical practice, RTX was initially used to treat non-lymphoma Hodgkin's before being extended to autoimmune diseases [24–26]. To investigate the effectiveness of RTX in individuals with IMN, we performed a meta-analysis.

## 2. Materials and Methods

### 2.1. Inclusion Criteria

The types of study design in published studies on the effectiveness of RTX for treating IMN were included.

### 2.2. Exclusion Criteria

The studies that include the animal experiments were not included.

### 2.3. Participant Selection

IMN patients without other systemic diseases were enrolled in this study.

### 2.4. Interventions Types

The control team received various therapies for IMN patients, which includes immunosuppressive therapy. Accepted regimens include steroids/cyclophosphamide (CTX), calcineurin inhibitors, and B cell depletion, while the intervention team received RTX along with other medicines.

### 2.5. Outcome Measure Types

Outcome indicators for patients with IMN (indicators analyzed using RTX in combination with other therapies for IMN): (1) overall effectiveness; (2) serum creatinine; (3) ALB; (4) adverse effects. The literature included in this study used at least one of the above scales to assess outcome indicators.

### 2.6. Search Strategy

The China Biomedical Literature Database (CBM), PubMed, EMbase, Web of Science, CNKI, VIP, Cochrane Library, and WanFang databases are all retrieved by the computer. The search term is “Zoledronic Sodium” and “Osteoporotic” and “Compression Fractures” and “Percutaneous Kyphoplasty” or “Percutaneous Vertebralplasty.” From the library's founding until February 2022, searches were conducted. The specific steps of literature search are (1) search for relevant documents in the Chinese and English databases, read the title, abstract, and keywords, further identify the search terms for this study; (2) the English database search used “MeSH Terms” to identify the subject terms, searched using a combination of subject words and keywords.

### 2.7. Extraction of Data and Quality Evaluation

The abstract was initially screened, and after the initial screening, the literature screening results were obtained by reading the full text, and the process was completed independently by 2 researchers. Exchange screening results, discuss dissenting literature or consult a third researcher until the results are agreed upon. The information extracted from the data includes basic information about the literature, type of study, study object, sample size, intervention content, and outcome measures.

### 2.8. Statistical Analysis

The review manager program was used to carry out this meta-analysis (RevMan). Effects are combined: The research's outcome metrics all are measured data, and the tools used to evaluate are different. There are differences between scores. Therefore, the standardized mean difference (SMD) is used (and 95% letters to the zone (confidence interval, CI) as an indicator of effect. Heterogeneity test: chi-square tests are used to determine whether there is heterogeneity between studies, if *P* > 0.1, *I*^2^ < 50%. The associated research was claimed to be more homogeneous, proceed with a fixed-effects model meta-analyses, if *P* < 0.1, *I*^2^ ≥ 50%. Heterogeneity was indicated in the included studies, analyze heterogeneous sources, if there is no clinical heterogeneity, a random-effects model is used for meta-analyses. Furthermore, possible differences in qualitative factors were subgroup analyzed.

## 3. Results

### 3.1. Detailed Information of the Included Studies

Six hundred seventy-seven citations were found using the search method. Identical research was eliminated, and then 355 articles were examined using the abstract and title. The full texts of 15 articles were then examined. Seven records were eliminated after a comprehensive text analysis due to data mismatch (*n* = 2) and missing data (*n* = 5). In the end, our meta-analysis included 8 studies [6–13] (Table 1). This procedure is depicted in the PRISMA statement flow chart (Figure 1).

### 3.2. Test group's Overall Effective Rate Was Substantially Greater Than the Control Group's

The combined effectiveness rate of the test category and the control category was reported in 6 investigations. The test group's overall effective rate was substantially greater than the control group's (OR: 1.37; 95% CI: 1.07, 1.76; *P* = 0.01, Figure 2). Due to the large degree of heterogeneity in the outcomes of all of these trials, a sensitivity analysis was carried out (Figure 3). RTX significantly raises the level of total effective rate in IMN patients when compared to the control group.

### 3.3. Blood Creatinine Levels of the Experimental Group and the Control Group Do Not Differ Statistically Significant

About 4 trials, the serum creatinine levels of the experimental group and the control group were recorded. The blood creatinine levels of the experimental group and the control group does not differ statistically significant, according to the meta-analysis (SMD: −6.87; 95% CI: −14.09, 0.35; *P* = 0.062, Figure 4). The overall serum creatinine level of the treatment group was lower than that of the control group, even though the meta-findings analyses were not statistically significant.

### 3.4. There Was No Large Discrepancy between the ALBs of the Experimental and Control Groups

The ALB of the test and control group were reported in 4 trials. According to meta-analysis, there was no large discrepancy between the ALBs of the experimental and control groups (Figure 5; SMD: 1.91; 95% CI: −0.31, 4.14, *P* = 0.092). The results of the meta-analysis were not statistically relevant, however, the treatment category had a greater total level of ALB than the control category.

### 3.5. Adverse Reactions

The negative effects on the test and control category were documented in 6 investigations. According to meta-analysis, the test group experienced considerably fewer negative reactions than the comparison group. Only the studies of Jun et al. [27] and the studies of Dahan et al. [33] exert the opposite results (OR: 0.56; 95% CI: 0.36, 0.90; *P* < 0.01; Figure 6).

### 3.6. Publication Bias

Despite the uneven distribution of the overall effective rate's funnel plot (Figure 7), Egger's test revealed that there was no probable publication bias (*P* = 0.256).

## 4. Discussion

A prevalent pathogenic form of NS in adults is called as MN, and it is characterized by the accumulation of immune complexes under the glomerular basement membrane and extensive basement membrane thickening [35, 36]. Men are more likely to experience it than women, and it affects those over 40. IMN and SMN are the two types, according to their genesis. It has been reported that about 80% of MN cases are related to renal function limitation (primary) and 20% are linked to additional systemic illnesses or vulnerabilities (secondary). The clinical onset of IMN is insidious, and the natural course of the disease varies greatly. Males are more likely to experience it than females do among middle-aged and elderly adults over the age of 40. Of those, NS affects over 80% [37] (clinical symptoms, such as large proteinuria, varying degrees of edema, hypoproteinemia, and hyperlipidemia), in which the incidence of thromboembolism is as high as 50–60% [38].

As a novel biological agent, RTX can target the pathogenesis of the disease and is more targeted than traditional immunosuppressive agents. RTX may be a promising alternative to glucocorticoid combined with immunosuppressive therapy. The effectiveness and efficacy of RTX in the management of IMN has recently been supported by numerous research findings. Numerous studies have shown that in patients refractory to CTX or calcineurin inhibitor therapy, 20–33% of patients who receive 2–4 cycles of RTX therapy experience complete remission, while 20–60% experience partial remission [39, 40], B cells depletion, and reduction of PLA2R antibodies predict resolution of proteinuria [41, 42].

Although MN can occur at any age, about 80–95% of patients are older than 30 years old, but in recent years, kidney biopsy data in our department show that the age of MN is younger. Propensity: a large number of studies have shown that the prognosis of IMN patients is related to the age at the time of renal biopsy. However, other studies have found that age is not associated with prognosis [43]. In MN, the incidence is higher in men, ranging from 1.1 : 1 to 5.4 : 1. Studies by Schieppati et al. showed that the male patients have a worse renal prognosis. Polanco et al. showed that the remission rate of renal disease in male IMN patients was significantly lower than that in female patients, but in multivariate Cox regression analysis, gender was not an independent predictor of renal disease remission [44]. However, other studies have shown that gender is not associated with remission of renal disease. Some authors believe that race is also one of the indicators that lead to differences in renal prognosis in IMN. Sprangers et al. compared Caucasian, African-American, and Hispanic IMN patients and found that non-white IMN patients had significantly lower rates of renal disease remission, but non-whites does not have a univariate Cox regression analysis. Significant statistical significance (*P* = 0.3), but only in multivariate Cox regression analysis (*P* = 0.04). Although other studies have shown that human leucocyte antigen may also be associated with the prognosis of patients with IMN [10], these results both lack the support of large-scale data, so the interpretation of these results still needs to be very cautious.

Hypoalbuminemia is very common in IMN patients, and about 60–70% of IMN patients have NS [45]. Plasma albumin levels and urinary protein levels are significantly correlated, so urinary protein excretion also exists in multivariate analysis and serum albumin levels may easily lead to collinearity problems, which can lead to biased results. Previous studies have found that serum albumin levels are associated with renal prognosis in patients with IMN, but some studies have found that no correlation between the two. Significant proteinuria is one of the main clinical features of patients with MN, and urinary protein levels are one of the most widely studied laboratory indicators. Most studies have shown that urinary protein levels at renal biopsy are significantly associated with prognosis in patients with IMN [46–48]. Studies have shown that the presence of NS in IMN patients or whether they can achieve remission of NS is an important indicator for predicting poor renal prognosis [49, 50]. However, the fluctuation of urine protein level is often very obvious, so it is very important to accurately measure the urine protein level. Several studies have shown that the presence of decreased renal function at the time of renal biopsy, manifested as increased serum creatinine, decreased creatinine clearance, or decreased estimated glomerular filtration rate, is a predictor of poor renal outcome in patients with IMN. Zuo et al. [51] showed that patients with CKD 3 at the time of renal biopsy had a 14-fold increased risk of adverse renal outcomes compared to the patients with CKD stages 1 and 2. Studies have shown that comorbid hypertension is an independent risk factor for poor renal prognosis in IMN patients [52–56]. In these studies, hypertension was defined as blood pressure greater than 140–150/90 mmHg or taking any antihypertensive medication. The study by Donadio et al. [57] showed that although baseline blood pressure was not related to renal prognosis if the mean blood pressure during follow-up was lower than 140/85 mmHg, the renal prognosis was significantly improved [58, 59].

This study utilized a total of 8 pieces of literature, with 230 individuals in the control group and 381 individuals in the experimental group. A meta-analysis revealed that RTX recipients with IMN had greater total effective rates than controls. The experimental group total effective rate was at a tolerable level according to meta-analysis (OR: 1.37; 95% CI: 1.07, 1.76; *P* < 0.01). According to the findings of the meta-analysis of serum creatinine and ALB, the experimental group serum creatinine and ALB does not meaningfully vary from those of the control group. [(SMD: −6.87; 95% CI: −14.09, 0.35; *P* = 0.062) and (SMD:1.91; 95% CI: −0.31,4.14; *P* = 0.092)]. When compared with the control, RTX reduced dramatically the adverse reactions in patients with IMN, according to the outcomes of the meta-analysis of ADR (OR: 0.56; 95% CI: 0.36, 0.90; *P* = 0.01). Egger's test revealed no potential publish bias even though the funnel plot of the overall effective frequency was asymmetrically distributed (*P* = 0.256).

The innovation and significance of this article was to show that RTX may be beneficial for individuals with IMN. The limitations of this systematic review are: only Chinese and English literature were searched, no other language literature was obtained, and there may be incomplete research inclusion and bias in selection. Therefore, we should be objective about some of the results of this meta-analysis.

## 5. Conclusion

As indicated by the overall effective rate, serum creatinine, ALB, and side effects, the findings of this study imply that RTX may be beneficial for individuals with IMN; however, these findings still need to be confirmed by other high-quality trials.

## Figures and Tables

**Figure 1:** PRISMA statement flow chart.

**Figure 2:** Forest plot of the total effective rate.

**Figure 3:** Sensitivity analysis of the total effective rate.

**Figure 4:** Forest plot of the serum creatinine.

**Figure 5:** Forest plot of the ALB.

**Figure 6:** Forest plot of the adverse reactions.

**Figure 7:** Funnel plot of the total effective rate.

**Table 1:** Basic characteristics of the included studies.

References	Sample size (T/C)	Men/women	Age (years) (mean ± SD) (T/C)	T	C	Main outcomes
Xu et al. [27]	36/36	45/27	47.75 ± 11.05/48.22 ± 10.14	RTX + methylprednisolone	Methylprednisolone	Total effective rate, ALB, adverse reactions
Liu et al. [28]	62/87	109/38	54.2 ± 13.4/51.9 ± 10.5	RTX + rormone	Tacrolimus + rormone	Total effective rate, serum creatinine, ALB, adverse reactions
Zhang et al. [29]	38/38	48/28	42.31 ± 2.16/42.28 ± 2.17	RTX + methylprednisolone	Tripterygium glycosides	Total effective rate, serum creatinine
Xu [30]	17/18	23/12	48.71 ± 13.67/50.28 ± 8.14	RTX	Cyclophosphamide + rormone	Total effective rate, serum creatinine, ALB
Zhu et al. [31]	26/41	50/17	41.73 ± 14.89/44.34 ± 10.57	RTX + tacrolimus	Tacrolimus	Serum creatinine, ALB, adverse reactions
van den Brand et al. [32]	100/103	148/55	51.5 ± 15.9/55.3 ± 12.7	RTX	Cyclophosphamide + rormone	Adverse reactions
Dahan et al. [33]	37/38	52/23	53.0/58.5	RTX + NIAT	NIAT	Total effective rate, adverse reactions
Fervenza et al. [34]	65/65	100/30	51.9 ± 12.6/52.2 ± 12.4	RTX	Cyclosporine	Total effective rate, adverse reactions

T: trial group; C: control group.

## Data Availability

Data supporting this research article are available from the corresponding author or first author on reasonable request.
